# Clinical Significance of Inflammatory Factors, Osteocalcin, and Matrix Metalloproteinase-8 in Gingival Crevicular Fluid in Drug Treatment of Severe Periodontitis

**DOI:** 10.1155/2022/8825540

**Published:** 2022-07-09

**Authors:** Jinxing Gao, Wenjun Shui, Lei Ren

**Affiliations:** ^1^Department of Stomatology, Center for Plastic & Reconstructive Surgery, Zhejiang Provincial People's Hospital (Affiliated People's Hospital, Hangzhou Medical College), Hangzhou 310014, Zhejiang, China; ^2^Department of Stomatology, Hangzhou Ruli Medical Beauty Hospital, Hangzhou 310014, Zhejiang, China; ^3^Department of Stomatology, Hangzhou Meilai Medical Beauty Hospital, Hangzhou 310014, Zhejiang, China

## Abstract

Whether gingival crevicular fluid (GCF) indexes in patients with severe periodontitis affect the efficacy of drug treatment was a new direction of recent research. At present, there were few studies on the effects of inflammatory indicators, BGP, and MMP-8 levels in GCF on the efficacy of drug treatment in such patients. So the purpose of this study was to observe the changes in osteocalcin (BGP), matrix metalloproteinase-8 (MMP-8), and inflammatory indexes levels in GCF of patients with severe periodontitis. The correlation between the above indexes and the effect of drug treatment in the patients was analyzed, in order to provide guidance for improving the clinical curative effect of severe periodontitis. A retrospective analysis was conducted to collect the baseline data of patients with severe periodontitis who were treated with Minocycline Hydrochloride Ointment in our hospital. The inflammatory indicators, BGP, and MMP-8 levels in GCF were analyzed before drug treatment, and the treatment effect on the patients was counted. Logistic regression was used to analyze the correlation between BGP, MMP-8, and inflammatory indicators levels in GCF and the drug treatment effect on the patients. After statistical analysis, we found that the response rate was 69% and the inefficiency was 31%. There were no significant differences in C-reactive protein (CRP) and tumor necrosis factor-*α* (TNF-*α*) levels between the inefficacy group and efficacy group (*P* > 0.05). Compared with the efficacy group, the levels of interleukin-6 (IL-6), interleukin-1*β* (IL-1*β*), interleukin-8 (IL-8), BGP, and MMP-8 were increased in the inefficacy group. High levels of IL-6, IL-1*β*, IL-8, BGP, and MMP-8 were associated with ineffective drug treatment in patients with severe periodontitis (all OR >1 and *P* < 0.05). Levels of IL-6, IL-1*β*, IL-8, BGP, and MMP-8 predicted that the AUCs of drug treatment failure in patients with severe periodontitis were all greater than 0.7, which were 1.398, 1.458, 1.244, 1.012, and 1.012, respectively. From this, we can conclude that increased levels of BGP, MMP-8, and inflammatory indicators such as IL-6, IL-1*β,* and IL-8 in GCF would increase the risk of ineffective drug treatment in patients with severe periodontitis. The clinical treatment plan could be adjusted according to the levels of the above indicators in GCF to improve the effectiveness of drug treatment in patients.

## 1. Introduction

Periodontitis is a kind of periodontal tissue chronic inflammation, caused by bacteria in dental plaque infringement of periodontal tissue and can lead to swollen gums, periodontal patient's bag overflow pus, loose teeth, etc. [1, 2]. Periodontitis is classified into mild, moderate, and severe periodontitis. Severe periodontitis inflammation is the most obvious, with a periodontal pocket depth greater than 6 mm, attachment loss of more than 5 mm, alveolar bone absorption exceeding 1/2 root length, multiple teeth bifurcation lesions, tooth loosening, and displacement [3]. Severe periodontitis seriously damages the oral health of patients. At present, the drug (minocycline hydrochloride) is widely used in the treatment of this disease, which can achieve long-term antibacterial and anti-inflammatory effects. However, after the end of the treatment cycle, there are still some patients with gum or alveolar bone damage, tooth loss, and other adverse conditions, resulting in frustrated efficacy. Therefore, how to improve the effectiveness of drug therapy and promote rehabilitation is an urgent problem for clinicians. It is of guiding significance to find out the factors influencing the therapeutic effect of severe periodontitis and adjust the treatment plan according to the factors. Previous studies generally focused on the drug treatment of severe periodontitis, but little attention was paid to the reasons affecting the efficacy of drug treatment, and the improvement of the efficacy of drug treatment was also stagnant. Therefore, this study attempted to explore the relevant indicators that may affect the therapeutic effect of drugs for severe periodontitis. Gingival Crevicular fluid (GCF) refers to the exudate of gingival tissue in the gingival sulci [4]. The liquid contains a variety of substances that reflect the pathophysiological status of periodontal tissue, among which inflammatory indicators are indicators reflecting the inflammatory state, osteocalcin promotes bone absorption, and MMP-8 is a proteolytic enzyme. These three indicators are closely related to periodontal tissue or bone destruction [5–7]. Therefore, it is speculated that inflammatory indicators, BGP, and MMP-8 levels in GCF may affect the efficacy of drug treatment for severe periodontitis, but there are few studies on this. Therefore, this study aimed to analyze the correlation between inflammation indexes, BGP, and MMP-8 in GCF and drug treatment effect in patients with severe periodontitis and to provide guidance for clinical improvement of drug efficacy in severe periodontitis.

## 2. Materials and Methods

### 2.1. Patients with Source

The technical roadmap of this study is shown in Figure 1. The baseline data of patients with severe periodontitis who received treatment (Minocycline Hydrochloride Ointment) in our hospital from January 2020 to January 2022, as well as the inflammatory indicators, BGP, and MMP-8 levels in GCF before treatment, were retrospectively collected. Inclusion criteria were as follows: (1) it met the clinical diagnostic criteria of severe periodontitis [8]; (2) chronic periodontitis; (3) has not received any medical treatment for the disease within the last 3 months; and (4) the baseline data and the inflammatory indicators, BGP, and MMP-8 in GCF before treatment were complete. Exclusion criteria were as follows: (1) allergic reaction to drugs used in this study; (2) oral diseases other than periodontitis; and (3) complicated infectious diseases. One hundred cases were chosen, 42 females and 58 males. Thirty-seven patients have been smokers and 21 had hypertension. The mean age, the mean course of the disease, and the mean body mass index were (48.47 ± 4.61) years, (3.61 ± 1.09) years, and (22.59 ± 2.29) kg/m^2^, respectively.

### 2.2. Material Collection

Medical records of patients were reviewed and clinical data were collected, including (1) baseline data: gender, smoking history, history of hypertension, age, course of the disease, and body mass index; (2) the inflammation indicators: CRP, IL-6, IL-1*β*, IL-8, and TNF-*α* in GCF; and (3) the levels of BGP and MMP-8 in GCF.

### 2.3. Efficacy Evaluation Criteria and Grouping

Evaluation criteria for the efficacy of drug therapy for severe periodontitis [9]: inefficacy was defined as no change in clinical symptoms and periodontal pocket depth or even replacement of treatment methods. Improvement was defined as partial disappearance of clinical symptoms, improvement of tooth loosening, periodontal pocket depth of 2-3 mm, and significant improvement of chewing function. A significant effect was defined as complete disappearance of clinical symptoms, periodontal pocket depth less than 2 mm, and return to normal masticatory function. The number of effective cases was the sum of the number of improvement cases and the number of significant effect cases. Patients assessed as “inefficacy” were included in the inefficacy group, and patients assessed as “improvement” or “significant effect” were included in the efficacy group.

### 2.4. Therapeutic Method

All patients were treated with minocycline hydrochloride (Sunstar INC., Approval No. H20150106, specification: 0.5 g *∗* 5 tablets) after basic treatment. Basic treatment: health education was first given to patients, and then subgingival curettage or supragingival scaling was used to remove calculus according to the location of calculus distribution. Drug treatment: the periodontal pocket was filled with Minocycline Hydrochloride Ointment, once a week, for consecutive 4 weeks.

### 2.5. Index Detection Method

Before drug treatment, patients were instructed to gargle with water, remove their gingival plaque and calculus, and collect GCF with a sterile filter paper strip weighing method. The GCF was centrifuged for 10 min at a speed of 10000 r/min to detect the levels of inflammatory indicators (including CRP, IL-6, IL-1*β*, IL-8, and TNF-*α*), BGP, and MMP-8. The CRP level was detected by the automatic biochemical analyzer BK-280 200. The levels of L-6, IL-1*β*, IL-8, TNF-*α*, and MMP-8 were detected by the DNM-9606 ELISA analyzer and its matching kit (Beijing Pulang New Technology Co., LTD.), and BGP was detected by electrochemiluminescence. All testing operations were conducted strictly following the kit instructions for the test instrument.

### 2.6. Statistical Methods

Statistical analyses of the data of this study were implemented in SPSS 19.0 software. The data belonging to measurement type and conforming to normal distribution were represented by “$\bar{x}$ ± *s*” and analyzed by *t*-test. Discontinuous data use cases or percentages, using chi-square test; logistic regression was used to find the correlation between inflammation indexes, BGP, and MMP-8 in GCF and drug treatment effect of patients. ROC curve was developed to evaluate the predictive value of inflammation indexes, BGP, and MMP-8 in GCF for drug treatment. The test level was *α* = 0.05.

## 3. Results

### 3.1. Baseline Data of Inefficacy Treatment Patients and Efficacy Treatment Patients

According to statistics, 69 cases (69%) of 100 patients were treated effectively, while 31 cases (31%) were not. Comparison of gender, smoking history, history of hypertension, age, course of the disease, and body mass index between inefficacy and efficacy groups showed *P* > 0.05. This part of data is shown in Table 1 and Figures 2 and 3.

### 3.2. Inflammatory Indexes, BGP, and MMP-8 Levels in GCF of Patients with Inefficacy Treatment and Efficacy Treatment

The CRP level and TNF-*α*level of the inefficacy group and efficacy group were compared (*P* > 0.05). Compared with the efficacy group, the levels of IL-6, IL-1*β*, IL-8, BGP, and MMP-8 of the inefficacy group were increased. This part of data is shown in Table 2 and Figures 3 and 4.

### 3.3. Logistic Regression Analysis of the Effect of IL-6, IL-1*β*, IL-8, BGP, and MMP-8 on Drug Treatment in Patients with Severe Periodontitis

The effect of drug treatment was taken as the dependent variable (1 = inefficacy; 0 = efficacy group), IL-6, IL-1*β*, IL-8, BGP, and MMP-8 levels were taken as independent variables. The logistic regression analysis was conducted, and it was concluded that high levels of IL-6, IL-1*β*, IL-8, BGP, and MMP-8 were associated with ineffective drug treatment in patients with severe periodontitis (all OR >1, *P* < 0.05). This part of data is shown in Table 3.

### 3.4. The Predictive Efficacy of IL-6, IL-1*β*, IL-8, BGP, and MMP-8 Levels in Severe Periodontitis Patients with Inefficacy Treatment

ROC curve was made by taking the effect of drug treatment as the status variable (1 = inefficacy; 0 = efficacy group) and Il-6, IL-1*β*, IL-8, BGP, and MMP-8 levels as the test variables (Figure 5). The results indicated that the AUCs of IL-6, IL-1*β*, IL-8, BGP, and MMP-8 levels in predicting drug treatment failure in patients with severe periodontitis were all greater than 0.7, indicating that the above indexes had a certain predictive value for drug treatment failure severe periodontitis, and the best predictive value could be obtained when the index reaches the optimal truncation value. This part of data is shown in Table 4.

## 4. Discussion

Periodontitis patients had periodontal tissue destruction, alveolar bone absorption, and periodontal attachment loss, and the oral microbes attached to the tooth surface and accumulated in the gingival groove, resulting in periodontal ecological environment disorders, resulting in gingival bleeding, dental plaque, and bacteria increase.

For the clinical treatment of severe periodontitis, the antimicrobial treatment way after foundation treatment was used more. Minocycline hydrochloride was used in the treatment of periodontitis, with strong bacteriostatic action (better than tetracycline), and it could effectively inhibit a variety of pathogenic bacteria such as *Staphylococcus aureus* and streptococcus, to reduce inflammation reaction [10]. However, there were still some patients with no improvement or even aggravation of symptoms and reduced quality of life after minocycline hydrochloride treatment. Therefore, it was of great significance to explore the factors influencing the therapeutic effect of drugs for the clinical treatment of severe periodontitis.

According to the results and data of this study, 100 patients with severe periodontitis regularly received minocycline hydrochloride based on basic treatment, and a total of 31 patients were ineffective, with an incidence of ineffective treatment of 31%, similar to the results of related studies [11]. Based on the data from this study, in contrast to patients with effective treatment, the levels of IL-6, IL-1*β*, IL-8, BGP, and MMP-8 in patients with ineffective treatment went up, suggesting that IL-6, IL-1*β*, IL-8, BGP, and MMP-8 were abnormally high in GCF in patients with severe periodontitis who failed drug treatment. Further logistic regression analysis suggested that high levels of IL-6, IL-1*β*, IL-8, BGP, and MMP-8 in GCF were associated with drug treatment failure in patients with severe periodontitis, suggesting that high levels of IL-6, IL-1*β*, IL-8, BGP, and MMP-8 would lead to increased risk of treatment failure in patients with severe periodontitis. The reasons were analyzed as follows: (1) as periodontitis was the periodontal tissue of the local inflammatory bowel disease, periodontal pathogens and lipopolysaccharide metabolites induced local inflammation and tissue destruction. At the same time, they also stimulate the host and activation of inflammatory cells and immune cells, which triggered systemic inflammation and immune response, leading to upregulation of inflammatory mediators' level and acute phase proteins level [12]. Il-6, IL-1*β*, and IL-8 were all inflammatory mediators that regulated the immune response in the host body to microbial infection and played a central role in the destruction of periodontal tissues [13–15]. Inflammatory indicators such as IL-6, IL-1*β*, and IL-8 with an abnormal upward trend would aggravate the injury degree of vascular endothelial cells and further aggravate the inflammatory response of periodontal tissues, which may reduce the effect of drug treatment and increase the risk of treatment failure. (2) BGP was a hormone-like peptide mainly expressed by osteoblasts, which could promote bone resorption and reflect bone metabolism [16]. The abnormal increase of BGP in GCF in patients with severe periodontitis indicated severe alveolar bone damage, which may reduce the effect of drug treatment and increase the probability of ineffective treatment. It was consistent with relevant research results [17,18]. (3) MMP-8 was a lytic enzyme, mainly secreted by inflammatory exudate cells, which could degrade extracellular matrix and was a major participant in dissolved proteins in periodontal tissue destruction [19]. MMP-8 had an inflammatory effect on the occurrence and development of periodontitis and could degrade the extracellular matrix directly or indirectly, thereby damaging periodontal tissues [20]. The release of MMP-8 in GCF increased, and patients with severe periodontitis experienced aggravated inflammatory response and severe destruction of periodontal tissue, leading to an increased risk of ineffective treatment. Relevant studies had shown that the level of MMP-8 in GCF was closely related to the severity of chronic periodontitis [21, 22]. The higher the MMP-8 level, the greater the severity of chronic periodontitis, which to some extent reduced the effectiveness of drug treatment and increased the risk of treatment failure. To further clarify the relationship between the content of IL-6, IL-1*β*, IL-8, BGP, and MMP-8 in GCF and the drug's therapeutic effect on severe periodontitis, our research team has drawn the ROC curve. Based on the analysis, we infer that the levels of IL-6, IL-1*β*, IL-8, BGP, and MMP-8 in GCF were predictive of the failure of drug therapy for severe periodontitis (AUC >0.7). These results indicated that the levels of IL-6, IL-1*β*, IL-8, BGP, and MMP-8 in GCF were associated with the failure of drug treatment for severe periodontitis and could be used as a risk predictor for predicting the failure of drug treatment for severe periodontitis.

## 5. Strengths and Limitations

This study was the first to analyze the correlation between the BGP, MMP-8, and inflammatory indicators (including IL-6, IL-1*β*, and IL-8) in GCF and the drug treatment effect in patients with severe periodontitis, which could provide guidance for improving drug efficacy of severe periodontitis in clinic. However, there were some deficiencies in this study, for example, the selection of study samples was limited, and the sampling of GCF was affected by a variety of complex factors (including age and the location of the sampled teeth), which might lead to a certain bias in the study results. Therefore, the samples should be expanded in future studies to further confirm the relationship between the inflammatory indexes, BGP, and MMP-8 in GCF and the therapeutic effect of severe periodontitis.

## 6. Conclusions

To sum up, increased levels of BGP, MMP-8, and inflammatory indicators such as IL-6, IL-1*β,* and IL-8 in GCF would increase the risk of ineffective drug treatment in patients with severe periodontitis. The clinical treatment plan could be adjusted according to the levels of the above indicators in GCF to improve the effectiveness of drug treatment in patients.

## Figures and Tables

**Figure 1:** The technical roadmap of this study.

**Figure 2:** Gender, smoking history, and hypertension history.

**Figure 3:** Age, disease course, body mass index, CRP, and TNF-*α.*

**Figure 4:** IL-6, IL-1*β*, IL-8, BGP, and MMP-8. Note: ^*∗*^means *P* < 0.05.

**Figure 5:** ROC curve.

**Table 1:** Comparison of baseline data of inefficacy treatment patients and efficacy treatment patients.

Group	Gender (male/female)	Smoking history (yes/no)	History of hypertension (yes/no)	Age (years)	A course of disease (years)	Body mass index (kg/m^2^)
Inefficacy group (*n* = 31)	(19/12)	(13/18)	(6/25)	48.37 ± 4.42	3.54 ± 1.15	22.55 ± 2.39
Efficacy group (*n* = 69)	(39/30)	(24/45)	(15/54)	48.56 ± 4.79	3.68 ± 1.03	22.63 ± 2.18
t/*χ*^2^	0.200	0.469	0.073	0.188	0.581	0.160
*P*	0.655	0.493	0.787	0.851	0.563	0.874

**Table 2:** Comparison of inflammatory indexes, BGP, and MMP-8 levels in GCF of patients with inefficacy treatment and efficacy treatment.

Indexes	Inefficacy group (*n* = 31)	Efficacy group (*n* = 69)	*t*	*P*
CRP (mg/L)	4.07 ± 1.14	4.26 ± 1.22	0.735	0.464
IL-6 (*μ*g/L)	11.02 ± 2.24	8.39 ± 2.45	5.094	<0.001
IL-1*β* (*μ*g/L)	9.85 ± 2.69	7.21 ± 2.23	5.130	<0.001
IL-8 (*μ*g/L)	15.39 ± 3.40	12.28 ± 3.44	4.196	0.003
TNF-*α* (pg/mL)	52.68 ± 11.87	49.37 ± 10.21	1.425	0.157
BGP (mg/*μ*L)	398.27 ± 51.13	352.91 ± 65.23	3.425	<0.001
MMP-8 (ng/mL)	334.54 ± 63.43	269.14 ± 66.10	4.632	<0.001

**Table 3:** Logistic regression analysis of the effect of IL-6, IL-1*β*, IL-8, BGP, and MMP-8 on drug treatment effect in patients with severe periodontitis.

Variable	*β*	Se	Wald *χ*^2^	*P*	OR	95% confidence interval	
						Lower limit	Upper limit
IL-6	0.335	0.141	5.681	0.017	1.398	1.061	1.842
IL-1*β*	0.377	0.160	5.587	0.018	1.458	1.067	1.994
IL-8	0.218	0.105	4.324	0.038	1.244	1.013	1.527
BGP	0.012	0.005	4.790	0.029	1.012	1.001	1.023
MMP-8	0.012	0.005	5.522	0.019	1.012	1.002	1.023

**Table 4:** The predictive efficacy of IL-6, IL-1*β*, IL-8, BGP, and MMP-8 levels in severe periodontitis patients with inefficacy treatment.

Indexes	AUC (95% CI)	Standard error	*P*	Optimum truncation value	Sensitivity	Specificity	Maximum index
IL-6	0.779 (0.683–0.876)	0.049	<0.001	9.285	0.903	0.609	0.512
IL-1*β*	0.759 (0.655–0.862)	0.053	<0.001	8.060	0.774	0.638	0.412
IL-8	0.758 (0.653–0.863)	0.054	<0.001	15.275	0.645	0.812	0.457
BGP	0.701 (0.595–0.806)	0.054	0.001	340.18	0.871	0.493	0.364
MMP-8	0.766 (0.666–0.866)	0.051	<0.001	284.165	0.871	0.638	0.509

## Data Availability

The data used to support the findings of this study are available from the corresponding author upon request.
